# Connectivity Index of Generalized Uncertain Graph

**DOI:** 10.1155/2022/4571530

**Published:** 2022-05-23

**Authors:** Jinchan Wang, Xiulian Gao, Xiaoshuang Zhou, Changyou Guo, Xiuling Yin

**Affiliations:** ^1^School of Mathematics and Big Data, Dezhou University, Dezhou 253023, China; ^2^School of Information Management, Dezhou University, Dezhou 253023, China

## Abstract

In the application of classical graph theory, there always are various indeterministic factors. This study studies the indeterministic factors in the connected graph by employing the uncertainty theory. First, this study puts forward two concepts: generalized uncertain graph and its connectivity index. Second, it presents a new algorithm to compute the connectivity index of an uncertain graph and generalized uncertain graph and verify this algorithm with typical examples. In addition, it proposes the definition and algorithm of *α*-connectivity index of generalized uncertain graph and verifies the stability and efficiency of this new algorithm by employing numerical experiments.

## 1. Introduction

In graph theory, the connectivity graph is a fundamental concept. Many phenomena in the real life can be conveniently described as the graphical problems, which are formed by the “points” and the “lines.” For example, a roadmap can be interpreted as a graph, the vertices are the junctions, and an edge is the stretch of road from one junction to the next [1]. Graph theory is an important branch of operation research, and it is a young but rapidly maturing subject. Graph theory originated in the eighteenth century. Euler solved the first real problem (seven bridges of Königsberg) using graph theory in 1736 [2, 3], which thereby made him a founder of graph theory.

The information of edges and vertices is completely deterministic in traditional graph theory. However, in applications, due to the complexity of the system, uncertain factors in the graph may appear and produce a new situation. For example, the optimal objective cannot be easily formulated if the weight of the edges is uncertain in some shortest path problems [4], and the classical algorithms fail to solve shortest path problems. Whether two vertices are connected by an edge cannot be accurately determined in real life, which results in the failure of proving the properties of uncertain graph by the classical method. To cope with the above situation, the concept of uncertain graph was proposed in 2011 in a reference [5].

Sometimes, whether some vertices exist cannot be completely determined and the information of edges cannot be completely determined. For example, in cloud computing networks, the vertices could represent data centers, with edges representing that the two data centers participate in the calculation at the same time. The vertices and the edges in cloud computing networks both have indeterminacy. As a result, it cannot be fully determined whether the graph is connected.

Generally, when we apply probability theory, the exact probability distribution has to be known. However, the probability distribution does not exist in some observational data of small samples. In this case, we must predict the data based on the experience of experts. To properly use empirical data, Professor Liu proposed the uncertainty theory [6] and revised in [7]. In an uncertain environment, the uncertainty theory is a very powerful tool to solve the situations in which only empirical data can be employed.

Based on the work of [8], this study attempts to deal with the situation where the existence of vertices and edges cannot be completely determined. Reference [8] first presented the concepts of generalized uncertain graph and its connectivity index. The study is mainly to compute the connectivity index of the generalized uncertainty graph. This study puts forward a new algorithm to compute the connectivity index by the uncertainty theory.

There are five sections in the study. Section 1 is the introduction of this study. Section 2 introduces the relevant concepts and relevant properties of the uncertainty theory and graph theory. Section 3 briefly introduces an uncertain graph and puts forward a new algorithm to compute the connectivity index of uncertain graph and then verifies this algorithm with typical examples. Section 4 proposes a new algorithm of connectivity index of generalized uncertain graph based on the concepts of generalized uncertain graph and connectivity index and employs numerical experiments to verify the correctness of this new algorithm. Section 5 is the conclusion of the study.

## 2. Preliminaries

### 2.1. Main Theorem in Uncertainty Theory

Professor Liu Baoding established the uncertainty theory system [9] in 2007, which was revised and improved in 2010 [7]. Today, the uncertainty theory is a very important branch of mathematics.

This study will shortly present the main developments of uncertainty theory in multiple fields. Reference [10] presented the uncertainty process and defined the uncertainty differential equation. Reference [11] proposed uncertain programming. Reference [4] explored the shortest path problem that the weight of the edges is uncertain in 2011. Reference [12] explored the connectivity index of uncertain graph in 2013. In the next few years, Gao has discussed the cycle index [13, 14], regularity index [8], tree index [15], and *α*-connectivity index [16] of uncertain graph. Reference [17] discussed some properties of uncertain relations on a finite set in 2014. Reference [18] discussed the distribution function of the diameter in uncertain graph in 2014. There are four main axioms in the uncertainty theory: normality, duality, subadditivity, and product axiom [6, 9]. References [6] and [9, 19] give the concepts and conclusions about the uncertainty theory used in the study.

**Theorem 1 (see [19]).**

The events *ζ*_1_, *ζ*_2_,…, *ζ*_*n*_ are independent Boolean uncertain variables, i.e.,

(1) $$\begin{array}{c} \zeta_{i}=\left\{\begin{array}{c} 1\text{ if its uncertain measure is }\delta_{i},\\ 0\text{ if its uncertain measure is }1-\delta_{i}, \end{array}\right. \end{array}$$

for *i*=1,2,…, *n*, respectively. When *g* is a Boolean function, *ζ*=*g*(*ζ*_1_, *ζ*_2_,…, *ζ*_*n*_) is a Boolean uncertain variable such that:

(2) $$\begin{array}{c} Μ\left\{\zeta =1\right\}=\left\{\begin{array}{cc} \underset{g\left(\zeta_{1},\zeta_{2},\ldots ,\zeta_{n}\right)=1}{\sup}\underset{1\leq i\leq n}{\min}v_{i}\left(y_{i}\right), & \text{if}\underset{g\left(\zeta_{1},\zeta_{2},\ldots ,\zeta_{n}\right)=1}{\sup}\underset{1\leq i\leq n}{\min}v_{i}\left(y_{i}\right)<0.5,\\ 1-\underset{g\left(\zeta_{1},\zeta_{2},\cdots ,\zeta_{n}\right)=0}{\sup}\underset{1\leq i\leq n}{\min}v_{i}\left(y_{i}\right), & \text{if}\underset{g\left(\zeta_{1},\zeta_{2},\ldots ,\zeta_{n}\right)=1}{\sup}\underset{1\leq i\leq n}{\min}v_{i}\left(y_{i}\right)\geq 0.5, \end{array}\right. \end{array}$$

where *y*_*i*_ is the real number either 0 or 1, and *v*_*i*_ is defined as follows:

(3) $$\begin{array}{c} v_{i}\left(y_{i}\right)=\left\{\begin{array}{cc} \delta_{i} & \text{if }y_{i}=1,\\ 1-\delta_{i} & \text{if }y_{i}=0, \end{array}\right. \end{array}$$

for *i*=1,2,…, *n*, respectively.

### 2.2. Main Concepts and Terminologies of Classical Graph

This part will introduce the definition of graph and some main concepts of classical graph theory. At the same time, it will discuss the main theorems about graphs with some examples. The following basic terminology and concepts are from [17].

A graph *G* means a finite nonempty 2-element set, which consists of a set of vertices and a set of edges. The numbers of vertices of *G* are called the order, and the numbers of edges of *G* are called the size. A path is an alternating sequence of vertices and edges if no vertices are repeated. Two vertices are said to be connected if there exists a path between the two vertices in the graph. A connected graph *G* means that there exists one path between any two vertices.

**Definition 1 (see[17]).**

Let *G* be an n-order and m-size graph, *V*(*G*)={*v*_1_, *v*_2_,…, *v*_*n*_} be its vertices' set, and *E*(*G*)={*e*_1_, *e*_2_,…, *e*_*m*_} be its edges. The symplectic *n* × *n* matrix is the adjacency matrix of *G*:

(4) $$\begin{array}{c} A_{G}=\left(\begin{array}{cccc} \delta_{11} & \delta_{12} & \ldots & \delta_{1n}\\ \delta_{21} & \delta_{22} & \ldots & \delta_{2n}\\ \vdots & \vdots & \ldots & \vdots \\ \delta_{n1} & \delta_{n2} & \ldots & \delta_{nn} \end{array}\right), \end{array}$$

where $\delta_{ij}=\left\{\begin{array}{cc} 1 & \text{if }v_{i}v_{j}\in E\left(G\right),\\ 0 & \text{if }v_{i}v_{j}\notin E\left(G\right). \end{array}\right.$

**Example 1 .**

Figure 1 is a 4-order graph.

The adjacency matrix of Figure 1 is as follows:

(5) $$\begin{array}{c} \left(\begin{array}{cccc} 0 & 1 & 0 & 1\\ 1 & 0 & 1 & 0\\ 0 & 1 & 0 & 1\\ 1 & 0 & 1 & 0 \end{array}\right). \end{array}$$

There is a very important theorem in the classical graph theory, and it is a sufficient and necessary condition to verify whether the graph is a connected graph.

**Theorem 2 .**

If *G* is a n-order graph and its symplectic adjacency matrix is the *A*_*G*_, let *R* be the *n* × *n* matrix, where

(6) $$\begin{array}{c} R=I+A_{G}+A_{G}^{2}+A_{G}^{3}+\cdots +A_{G}^{n-1}. \end{array}$$

Then, *G* is a connected graph if and only if *R* > 0.

To analyze graphs and their properties with uncertainty factors, the fundamental concepts are given as follows.

**Definition 2 .**

If a symplectic adjacency matrix of the n-order graph is *A*_*G*_, the connectivity function of *G* is the following function:

(7) $$\begin{array}{c} C\left(A_{G}\right)=\left\{\begin{array}{cc} 1, & \text{if }I+A_{G}+A_{G}^{2}+A_{G}^{3}+\cdots +A_{G}^{n-1}>0,\\ 0, & \text{otherwise.} \end{array}\right. \end{array}$$

## 3. Uncertainty Graphs

### 3.1. Basic Concepts

Every vertex and edge of a graph is wholly determined. That is to say, the vertex and the edge either exist or do not exist in the classical graph theory. An *n*-order graph may be defined as a *n* × *n* symplectic adjacency matrix, and its elements are either 1 or 0. At the same time, the indeterminacy factor will absolutely occur in practical applications. To study this problem, [12] gave the concept of uncertain graph, which means all edges are independent and exist with uncertain measure. That is, the elements are no longer 1 or 0 in adjacency matrix, but a number in [0,1]. For instance, *δ*_*ij*_=0.65 represents that the uncertain measure is 0.65 about the edge existing between the two vertices, and the uncertain measure is 0.35 about the edge not existing between the two vertices.

**Definition 3 (see [12]).**

The *n*-order graph *G* is called an uncertain graph if its symplectic adjacency matrix is as follows:

(8) $$\begin{array}{c} A_{G}=\left(\begin{array}{cccc} \delta_{11} & \delta_{12} & \ldots & \delta_{1n}\\ \delta_{21} & \delta_{22} & \ldots & \delta_{2n}\\ \vdots & \vdots & \ldots & \vdots \\ \delta_{n1} & \delta_{n2} & \ldots & \delta_{nn} \end{array}\right), \end{array}$$

where *δ*_*ij*_ means the uncertain measure of the edge between vertexes *i* and *j*, for *i*, *j*=1,2,…, *n*, respectively.

It should be noted that *δ*_*ii*_=0(*i*=1,2,…, *n*) in the uncertain adjacency matrix. Besides, an uncertain adjacency matrix is symmetric if the uncertain graph is undirected; i e., *δ*_*ij*_=*δ*_*ji*_ for any *i* and *j*. Evidently, all the information of an uncertain graph may be contained in the symmetric adjacency matrix.

**Example 2 .**

An uncertain 4-order graph is as the following in Figure 2.

The symmetric adjacency matrix of Figure 2 is as follows:

(9) $$\begin{array}{c} \left(\begin{array}{cccc} 0 & 0.8 & 0.6 & 0.2\\ 0.8 & 0 & 0.4 & 0.7\\ 0.6 & 0.4 & 0 & 0.3\\ 0.2 & 0.7 & 0.3 & 0 \end{array}\right). \end{array}$$

We may know that the edge set of *G* is an uncertain Boolean variable set according to the definition of uncertain graph.

(10) $$\begin{array}{c} E\left(G\right)=\left\{\zeta_{12},\zeta_{13},\ldots ,\zeta_{1n},\zeta_{23},\ldots ,\zeta_{2n},\zeta_{34},\ldots ,\zeta_{3n},\ldots ,\zeta_{\left(n-1\right)n}\right\}, \end{array}$$

where Μ{*ζ*_*ij*_=1}=*δ*_*ij*_, for any 1 ≤ *i* < *j* ≤ *n*. For the sake of simplicity, we remove these edges *ζ*_*ij*_ satisfying Μ{*ζ*_*ij*_=1}=0 and denote as *E*(*G*)={*ζ*_1_, *ζ*_2_,…, *ζ*_*m*_}.

**Definition 4 (see [12]).**

Let *G* be an uncertain graph and *E*(*G*)={*ζ*_1_, *ζ*_2_,…, *ζ*_*m*_} be its edge set, and then, connectivity function of *G* may be denoted as follows:

(11) $$\begin{array}{c} \mathbb{C}\left(G\right)=\left\{\begin{array}{cc} 1, & \text{if }G\text{ is }a\text{ connected graph},\\ 0, & \text{otherwise.} \end{array}\right. \end{array}$$

Evidently, *ℂ*(*G*) is a Boolean function. We define the connectivity index of an uncertain graph *G* with *E*(*G*)={*ζ*_1_, *ζ*_2_,…, *ζ*_*m*_} as follows:

(12) $$\begin{array}{c} \partial \left(G\right)=Μ\left\{\mathbb{C}\left(G\right)=1\right\}. \end{array}$$

In other words, the connectivity index is the uncertain measure of the connected graph.

The key is how to obtain the connectivity index in a given uncertain graph. A theorem is proposed to deal with this problem.

**Theorem 3 .**

Let *G* be an n-order uncertain graph with a symmetric adjacency matrix as follows:

(13) $$\begin{array}{c} A_{G}=\left(\begin{array}{cccc} \delta_{11} & \delta_{12} & \ldots & \delta_{1n}\\ \delta_{21} & \delta_{22} & \ldots & \delta_{2n}\\ \vdots & \vdots & \ldots & \vdots \\ \delta_{n1} & \delta_{n2} & \ldots & \delta_{nn} \end{array}\right). \end{array}$$

The connectivity index of *G* is the formula (14) if all edges are independent.

(14) $$\begin{array}{c} \partial \left(G\right)=\left\{\begin{array}{cc} \underset{\mathbb{C}\left(Y\right)=1}{\sup}\underset{1\leq i<j\leq n}{\min}\nu_{ij}\left(y_{ij}\right), & \text{if }\underset{\mathbb{C}\left(Y\right)=1}{\sup}\underset{1\leq i<j\leq n}{\min}\nu_{ij}\left(y_{ij}\right)<0.5,\\ 1-\underset{\mathbb{C}\left(Y\right)=0}{\sup}\underset{1\leq i<j\leq n}{\min}\nu_{ij}\left(y_{ij}\right), & \text{if }\underset{\mathbb{C}\left(Y\right)=1}{\sup}\underset{1\leq i<j\leq n}{\min}\nu_{ij}\left(y_{ij}\right)\geq 0.5, \end{array}\right. \end{array}$$

where *Y* is an uncertain symmetric matrix and its diagonal entries are zero, and *Y* is denoted as follows:

(15) $$\begin{array}{c} Y=\left(\begin{array}{cccc} y_{11} & y_{12} & \cdots & y_{1n}\\ y_{21} & y_{22} & \cdots & y_{2n}\\ \vdots & \vdots & \vdots & \vdots \\ y_{n1} & y_{n2} & \cdots & y_{nn} \end{array}\right), \end{array}$$

and *y*_*ij*_=*y*_*ji*_ is equal to either 0 or 1 and *y*_*ii*_=0, and *v*_*ij*_ is denoted as follows:

(16) $$\begin{array}{c} v_{ij}\left(y_{ij}\right)=\left\{\begin{array}{cc} \delta_{ij}, & \text{when }y_{ij}=1,\\ 1-\delta_{ij}, & \text{when }y_{ij}=0, \end{array}\right. \end{array}$$

for *i*=1,2,…, *n*; *j*=1,2,…, *n*, respectively, and

(17) $$\begin{array}{c} \mathbb{C}\left(Y\right)=\left\{\begin{array}{cc} 1, & \text{if }I+Y+Y^{2}+Y^{3}+\ldots +Y^{n-1}>0,\\ 0, & \text{otherwise.} \end{array}\right. \end{array}$$

**Proof**

Since *y*_*ij*_ is independent Boolean uncertain variables for any *i* and *j*, *Y* is the Boolean symmetric uncertain matrix. Therefore, we may get that the function *ℂ*(*Y*) is a Boolean function based on Definition 3. Therefore, according to Theorem 1, we have the following:

(18) $$\begin{array}{c} M\left\{\mathbb{C}\left(Y\right)=1\right\}=\left\{\begin{array}{cc} \underset{\mathbb{C}\left(Y\right)=1}{\sup}\underset{1\leq i<j\leq n}{\min}\nu_{ij}\left(y_{ij}\right), & \text{if }\underset{\mathbb{C}\left(Y\right)=1}{\sup}\underset{1\leq i<j\leq n}{\min}\nu_{ij}\left(y_{ij}\right)<0.5,\\ 1-\underset{\mathbb{C}\left(Y\right)=0}{\sup}\underset{1\leq i<j\leq n}{\min}\nu_{ij}\left(y_{ij}\right), & \text{if }\underset{\mathbb{C}\left(Y\right)=1}{\sup}\underset{1\leq i<j\leq n}{\min}\nu_{ij}\left(y_{ij}\right)\geq 0.5, \end{array}\right. \end{array}$$

where *Y* is the symmetric uncertain matrix as follows:

(19) $$\begin{array}{c} Y=\left(\begin{array}{cccc} y_{11} & y_{12} & \cdots & y_{1n}\\ y_{21} & y_{22} & \cdots & y_{2n}\\ \vdots & \vdots & \vdots & \vdots \\ y_{n1} & y_{n2} & \cdots & y_{nn} \end{array}\right), \end{array}$$

and *y*_*ij*_=*y*_*ji*_ is equal to either 0 or 1 and *y*_*ij*_=*y*_*ji*_, and *v*_*ij*_ is defined as follows:

(20) $$\begin{array}{c} v_{ij}\left(y_{ij}\right)=\left\{\begin{array}{cc} \delta_{ij}, & \text{when }y_{ij}=1,\\ 1-\delta_{ij}, & \text{when }y_{ij}=0, \end{array}\right. \end{array}$$

for any *i*, *j*. The connectivity index of an uncertain graph is the uncertain measure of connected graph according to Definition 4. Therefore, Theorem 2 has been proved.

However, the connectivity index is difficult to obtain from Theorem 1 as to other more complex graphs. A new theorem to compute the connectivity index will be given. First, some new definitions will be introduced in the following.

**Definition 5 .**

Assume *A*=(*a*_*ij*_) and *B*=(*b*_*ij*_) be all the *m* × *n* matrices. Then, the logic sum *A* ⊕ *B* is defined as follows:

(21) $$\begin{array}{c} A⊕B=\left(c_{ij}\right), \end{array}$$

where *c*_*ij*_=*a*_*ij*_∨*b*_*ij*_=max{*a*_*ij*_, *b*_*ij*_}.

**Definition 6 .**

Assume *A*=(*a*_*ij*_) be *m* × *k* matrix and *B*=(*b*_*ij*_) be *k* × *n* matrix. Then, the logic product *A*∘*B* is defined as follows:

(22) $$\begin{array}{c} A\circ B=\left(c_{ij}\right), \end{array}$$

where $c_{ij}=\vee_{p=1}^{k}\left(a_{ip}\wedge b_{pj}\right)=\underset{1\leq p\leq k}{\max}\left\{\min\left\{a_{ip},b_{pj}\right\}\right\}$.

**Definition 7 .**

Assume *A*=(*a*_*ij*_) be the *n* × *n* matrix. Then, the logic power *A*^(*k*)^ is defined as follows:

(23) $$\begin{array}{c} A^{\left(k\right)}=A^{\left(k-1\right)}\circ A, \end{array}$$

where I be the *n* × *n* unit matrix, *A*^(1)^=*A* and *A*^(0)^=*I*.

**Definition 8 .**

Let *G* be an n-order uncertain graph and its symmetric adjacency matrix be as follows:

(24) $$\begin{array}{c} A_{G}=\left(\begin{array}{cccc} \delta_{11} & \delta_{12} & \ldots & \delta_{1n}\\ \delta_{21} & \delta_{22} & \ldots & \delta_{2n}\\ \vdots & \vdots & \ldots & \vdots \\ \delta_{n1} & \delta_{n2} & \ldots & \delta_{nn} \end{array}\right). \end{array}$$

Then, the reachable measure matrix *P* of uncertain graph *G* is defined as follows:

(25) $$\begin{array}{c} P=I⊕A_{G}⊕A_{G}^{\left(2\right)}⊕A_{G}^{\left(3\right)}⊕\ldots ⊕A_{G}^{\left(n-1\right)}. \end{array}$$

**Theorem 4 .**

Let *G* be an n-order uncertain graph and its uncertain symmetric adjacency matrix be *A*_*G*_, and its reachable measure matrix be *P*, and then, the connectivity index of *G* is the smallest number in the reachable measure matrix *P*.

**Proof**

Since connectivity index of an uncertain graph is the uncertain measure of the connected graph based on Definition 4, a connected graph *G* is that any two vertices are connected in the graph *G*. That is, there exists at least a path between any two vertices in the graph *G*. Thus, we only need to prove that the element *δ*_*ij*_^(*k*)^ in *A*_*G*_^(*k*)^ is the uncertain measure that there exists at least a path whose length is *k* from the vertexes *i* to *j* in the graph *G*. In a *n*-order graph, the length of a path at most is *n* − 1. Then, we can know that Theorem 4 is the right according to the previous theorem and definition.

Now, we begin to prove the conclusion that the element *δ*_*ij*_^(*k*)^ in *A*_*G*_^(*k*)^ is the uncertain measure that there exists at least a path whose length is *k* from the vertexes *i* to *j* in the graph *G* using mathematical induction.

Obviously, the conclusion is correct when *k* = 0 or 1.

If *k* = 2, based on Definition 6 and Definition 7, we have the following:

(26) $$\begin{array}{c} \delta_{ij}^{\left(2\right)}=\overset{n}{\underset{l=1}{\vee }}\left(\delta_{il}\wedge \delta_{lj}\right), \end{array}$$

where *δ*_*il*_ represents that the edge *e*_*il*_ between vertexes *i* and *l* exists with uncertain measure *δ*_*il*_, and *δ*_*lj*_ represents that the edge *e*_*lj*_ between vertexes *l* and *j* exists with uncertain measure *δ*_*lj*_, and *δ*_*il*_∧*δ*_*lj*_ represents the uncertain measure that the two edges *e*_*il*_ and *e*_*lj*_ exist at the same time; i.e., *δ*_*il*_∧*δ*_*lj*_ represents the uncertain measure of the path whose length is 2 from the vertexes *i* to *j* via vertex *l*. So, ∨_*l*=1_^*n*^(*δ*_*il*_∧*δ*_*lj*_) represents the uncertain measure that there exists at least a path whose length is 2 from the vertexes *i* to *j*.

According to the above discussion, the conclusion is correct when *k* = 2.

Assume the conclusion is correct when *k* = *p*, and then, when *k* = *p* + 1, we have the following:

(27) $$\begin{array}{c} \delta_{ij}^{\left(p+1\right)}=\overset{n}{\underset{l=1}{\vee }}\left(\delta_{il}^{\left(p\right)}\wedge \delta_{lj}\right), \end{array}$$

where *δ*_*il*_^(*p*)^ represents the uncertain measure that there exists at least a path whose length is *p* from the vertexes *i* to *l* in the graph *G*, and *δ*_*lj*_ represents that the edge *e*_*lj*_ between vertexes *l* and *j* exists with uncertain measure *δ*_*lj*_, and *δ*_*il*_^(*p*)^∧*δ*_*lj*_ represents the uncertain measure that the path whose length is *p* from the vertexes *i* to *l* and edge *e*_*lj*_ exists at same time; i.e., *δ*_*il*_^(*p*)^∧*δ*_*lj*_ represents the uncertain measure of the path whose length is *p* + 1 from the vertexes *i* to *j* via vertex *l*. So, ∨_*l*=1_^*n*^(*δ*_*il*_^(*p*)^∧*δ*_*lj*_) represents the uncertain measure that there exists at least a path whose length is *p* + 1 from the vertexes *i* to *j*. Thus, the conclusion is correct when *k* = *p* + 1.

From what has been discussed above, the conclusion is correct, for *k*=0,1,2,…, *n* − 1, respectively. Therefore, Theorem 3 has been proved.

**Example 3 .**

Figure 2 illustrates the uncertain 4-order graph, and its symmetric adjacency matrix is as follows:

(28) $$\begin{array}{c} A_{G}=\left(\begin{array}{cccc} 0 & 0.8 & 0.6 & 0.2\\ 0.8 & 0 & 0.4 & 0.7\\ 0.6 & 0.4 & 0 & 0.3\\ 0.2 & 0.7 & 0.3 & 0 \end{array}\right). \end{array}$$

Now, we compute its connectivity index according to Theorem 3.

(29) $$\begin{array}{c} A_{G}^{\left(1\right)}=A_{G},\\ A_{G}^{\left(2\right)}=\left(\begin{array}{cccc} 0 & 0.8 & 0.6 & 0.2\\ 0.8 & 0 & 0.4 & 0.7\\ 0.6 & 0.4 & 0 & 0.3\\ 0.2 & 0.7 & 0.3 & 0 \end{array}\right)\circ \left(\begin{array}{cccc} 0 & 0.8 & 0.6 & 0.2\\ 0.8 & 0 & 0.4 & 0.7\\ 0.6 & 0.4 & 0 & 0.3\\ 0.2 & 0.7 & 0.3 & 0 \end{array}\right)=\left(\begin{array}{cccc} 0.8 & 0.4 & 0.4 & 0.7\\ 0.4 & 0.8 & 0.6 & 0.3\\ 0.4 & 0.6 & 0.6 & 0.4\\ 0.7 & 0.3 & 0.4 & 0.7 \end{array}\right),\\ A_{G}^{\left(3\right)}=\left(\begin{array}{cccc} 0.8 & 0.4 & 0.4 & 0.7\\ 0.4 & 0.8 & 0.6 & 0.3\\ 0.4 & 0.6 & 0.6 & 0.4\\ 0.7 & 0.3 & 0.4 & 0.7 \end{array}\right)\circ \left(\begin{array}{cccc} 0 & 0.8 & 0.6 & 0.2\\ 0.8 & 0 & 0.4 & 0.7\\ 0.6 & 0.4 & 0 & 0.3\\ 0.2 & 0.7 & 0.3 & 0 \end{array}\right)=\left(\begin{array}{cccc} 0.4 & 0.8 & 0.6 & 0.4\\ 0.8 & 0.4 & 0.4 & 0.7\\ 0.6 & 0.4 & 0.4 & 0.6\\ 0.4 & 0.7 & 0.6 & 0.3 \end{array}\right),\\ P=I\;⊕\;A_{G}^{\left(1\right)}\;⊕\;A_{G}^{\left(2\right)}\;⊕\;A_{G}^{\left(3\right)},\\ =\left(\begin{array}{cccc} 1 & 0 & 0 & 0\\ 0 & 1 & 0 & 0\\ 0 & 0 & 1 & 0\\ 0 & 0 & 0 & 1 \end{array}\right)⊕\left(\begin{array}{cccc} 0 & 0.8 & 0.6 & 0.2\\ 0.8 & 0 & 0.4 & 0.7\\ 0.6 & 0.4 & 0 & 0.3\\ 0.2 & 0.7 & 0.3 & 0 \end{array}\right)⊕\;\left(\begin{array}{cccc} 0.8 & 0.4 & 0.4 & 0.7\\ 0.4 & 0.8 & 0.6 & 0.3\\ 0.4 & 0.6 & 0.6 & 0.4\\ 0.7 & 0.3 & 0.4 & 0.7 \end{array}\right)\;⊕\;\left(\begin{array}{cccc} 0.4 & 0.8 & 0.6 & 0.4\\ 0.8 & 0.4 & 0.4 & 0.7\\ 0.6 & 0.4 & 0.4 & 0.6\\ 0.4 & 0.7 & 0.6 & 0.3 \end{array}\right)\\ =\left(\begin{array}{cccc} 1 & 0.8 & 0.6 & 0.7\\ 0.8 & 1 & 0.6 & 0.7\\ 0.6 & 0.6 & 1 & 0.6\\ 0.7 & 0.7 & 0.6 & 1 \end{array}\right). \end{array}$$

So, we can know that the connectivity index of the uncertain graph in Figure 2 is 0.6 according to Theorem 3.

In 2014, the distribution function of the diameter of uncertain graph is discussed in reference [18]. The diameter is an uncertain variable in uncertain graph since the existence of each edge is uncertain. The diameter is a fundamental concept in the graph theory, which means the maximal distance between any two vertices; that is, the diameter in determinate graph *G* =(*V, E*) is diam(*G*) =  $\underset{v_{i},v_{j}\in V}{\max}d\left(v_{i},v_{j}\right)$. Based on Theorem 3, the following conclusion can calculate the distribution function of the diameter in an uncertain graph.

**Corollary 1 .**

Let *G* be an uncertain n-order graph and its uncertain symmetric adjacency matrix be *A*_*G*_. Let the matrix *D* be described as follows:

(30) $$\begin{array}{c} D=I⊕A_{G}⊕A_{G}^{\left(2\right)}⊕A_{G}^{\left(3\right)}⊕\ldots ⊕A_{G}^{\left(k\right)}. \end{array}$$

Then, the uncertainty distribution of the diameter in the graph *G* is as follows:

(31) $$\begin{array}{c} M\left\{\text{diam}\left(G\right)\leq k\right\}=\underset{1\leq i,j\leq n}{\min}\left\{d_{ij}\right\}, \end{array}$$

where *k* (*k* ≤ *n* − 1) is a positive integer and *d*_*ij*_ is the element in *D*.

In the next section, the connectivity of generalized uncertain graph is investigated and analyzed.

## 4. Generalized Uncertainty Graphs

### 4.1. Basic Concepts and Algorithms

Not only whether an edge exists between two vertices cannot be completely determined but also whether some vertices exist cannot be completely determined in applications of traditional graph theory. In the study, the indeterministic factors are that whether vertices and edges exist is uncertain. If there are no historical data or experimental data, a random variable cannot be employed to describe this indeterministic factor. Often, we may consult experts and ask them to give a belief degree that the edge exists. The experience data are precisely the research category of uncertainty theory. Therefore, uncertain variable is employed to describe the indeterministic factor in this study.

**Definition 9 .**

A n-order graph is called a generalized uncertain graph if its symmetric adjacency matrix is as follows:

(32) $$\begin{array}{c} A_{G}=\left(\begin{array}{ccccc} 0 & \delta_{12} & \cdots & \delta_{1n} & \delta_{1}\\ \delta_{21} & 0 & \cdots & \delta_{2n} & \delta_{2}\\ \vdots & \vdots & \vdots & \vdots & \vdots \\ \delta_{n1} & \delta_{n2} & \cdots & 0 & \delta_{n}\\ \delta_{1} & \delta_{2} & \cdots & \delta_{n} & 0 \end{array}\right), \end{array}$$

where *δ*_*ij*_ represents the uncertain measure of edges and *δ*_*k*_ represents the uncertain measure of vertex.

It should be noted that there always are *δ*_*ii*_=0 in the generalized uncertain adjacency matrix.

From the above, we know that all the information of a generalized uncertain graph is contained in the adjacency matrix.

**Example 4 .**

Figure 3 is a generalized uncertain 4-order graph as follows.

The adjacency matrix of Figure 3 is as follows:

(33) $$\begin{array}{c} \left(\begin{array}{ccccc} 0 & 0.85 & 0.65 & 0.15 & 0.95\\ 0.85 & 0 & 0.45 & 0.75 & 0.35\\ 0.65 & 0.45 & 0 & 0.35 & 0.75\\ 0.15 & 0.75 & 0.35 & 0 & 0.65\\ 0.95 & 0.35 & 0.75 & 0.65 & 0 \end{array}\right). \end{array}$$

**Definition 10 .**

Suppose *G* is a generalized uncertain n-order graph, and its adjacency matrix is as follows:

(34) $$\begin{array}{c} A_{G}=\left(\begin{array}{ccccc} 0 & \delta_{12} & \cdots & \delta_{1n} & \delta_{1}\\ \delta_{21} & 0 & \cdots & \delta_{2n} & \delta_{2}\\ \vdots & \vdots & \vdots & \vdots & \vdots \\ \delta_{n1} & \delta_{n2} & \cdots & 0 & \delta_{n}\\ \delta_{1} & \delta_{2} & \cdots & \delta_{n} & 0 \end{array}\right), \end{array}$$

where *δ*_*ij*_ represents the uncertain measure of edges between two vertexes and *δ*_*k*_ represents the uncertain measure of vertex. The basic graph $\bar{G}$ of generalized uncertain graph *G* is defined as an uncertain graph with the following adjacency matrix:

(35) $$\begin{array}{c} B_{G}=\left(\begin{array}{cccc} \lambda_{11} & \lambda_{12} & \cdots & \lambda_{1n}\\ \lambda_{21} & \lambda_{22} & \cdots & \lambda_{2n}\\ \vdots & \vdots & \vdots & \vdots \\ \lambda_{n1} & \lambda_{n2} & \cdots & \lambda_{nn} \end{array}\right), \end{array}$$

where *λ*_*ij*_=min{*δ*_*ij*_, *δ*_*i*_, *δ*_*j*_}.

**Example 5 .**

Figure 4 is the basic graph of Figure 3.

The symmetric adjacency matrix of Figure 4 is as follows:

(36) $$\begin{array}{c} \left(\begin{array}{cccc} 0 & 0.35 & 0.65 & 0.15\\ 0.35 & 0 & 0.35 & 0.35\\ 0.65 & 0.35 & 0 & 0.35\\ 0.15 & 0.35 & 0.35 & 0 \end{array}\right). \end{array}$$

**Definition 11 .**

Suppose that *G* is a generalized uncertain graph with a symmetric adjacency matrix as follows:

(37) $$\begin{array}{c} A_{G}=\left(\begin{array}{ccccc} 0 & \delta_{12} & \cdots & \delta_{1n} & \delta_{1}\\ \delta_{21} & 0 & \cdots & \delta_{2n} & \delta_{2}\\ \vdots & \vdots & \vdots & \vdots & \vdots \\ \delta_{n1} & \delta_{n2} & \cdots & 0 & \delta_{n}\\ \delta_{1} & \delta_{2} & \cdots & \delta_{n} & 0 \end{array}\right). \end{array}$$

The connectivity function of *G* is expressed as follows:

(38) $$\begin{array}{c} \mathbb{C}\left(G\right)=\left\{\begin{array}{cc} 1, & \text{if graph }G\text{ is connected},\\ 0, & \text{otherwise.} \end{array}\right. \end{array}$$

From the above, we can know that *ℂ*(*G*) is a Boolean function. Thus, in a generalized uncertain graph *G* the connectivity index may be denoted as follows:

(39) $$\begin{array}{c} \partial \left(G\right)=M\left\{\mathbb{C}\left(G\right)=1\right\}. \end{array}$$

Namely, the connectivity index is the uncertain measure to which the generalized uncertain graph is connected.

Obviously, the connectivity index of a generalized uncertain graph is exactly equal to the connectivity index of its basic graph.

Based on some of the ideas that we have discussed above, we may know the connectivity index of a generalized uncertain graph, and then, we may compute the connectivity index of a generalized uncertain graph as follows.

**Step 1 .**

To write out the adjacency matrix of the generalized uncertain graph *G*.

**Step 2 .**

To compute the adjacency matrix of the basic graph $\bar{G}$ of the generalized uncertain graph *G*.

**Step 3 .**

To compute the connectivity index of the basic graph $\bar{G}$ of the generalized uncertain graph *G* according to Theorem 3, and thus, the connectivity index of generalized uncertain graph is obtained.

### 4.2. Examples

In this part, two examples are given to compute the connectivity index of a generalized uncertain graph.

**Example 6 .**

Figure 5 is a 2-order generalized uncertain graph *G* and the uncertain measure of edge is *a*, and the uncertain measure of vertices is *α* and *β* respectively.

In Figure 5, the connectivity index of *G* is the smallest number of *α*, *β*, and *a*.

**Example 7 .**

Figure 6 illustrates a 3-order uncertain graph *G*, and the uncertain measure of edges is 0.8, 0.7, and 0.6, respectively, and uncertain measure of vertices is 0.75, 0.9, and 0.8, respectively.

As Figure 6 illustrates a 3-order generalized uncertain graph (G), its basic graph is shown in Figure 7. In Figure 6, the connectivity index of (*G*) is 0.7 by Theorem 1.

**Example 8 .**

Figure 3 illustrates a 4-order generalized uncertain graph *G*, and the uncertain measure of its edges is 0.8, 0.7, 0.6, 0.4, 0.3, and 0.1, respectively, and the uncertain variables of its vertices are 0.9, 0.3, 0.7, and 0.6, respectively.

Because Figure 3 is a 4-order generalized uncertain graph, its basic graph is Figure 4, and the connectivity index of *G* in Figure 3 is 0.3 by Theorem 3.

### 4.3. *α*-Connectivity of Generalized Uncertain Graph

**Definition 12 .**

Let *G* be a generalized uncertain graph with a confidence level *α*. If the uncertain measure of an edge or vertex in *G* is not smaller than the confidence level *α*, the uncertain measure is mapped as 1, or the uncertain measure is replaced by 0. Thus, a sample subgraph of *G* can be obtained and the sample subgraph is referred to as fundamental subgraph about the confidence level *α*.

**Definition 13 .**

A generalized uncertain graph *G* is called *α*-connected if its fundamental subgraph about the confidence level *α* is connected.

According to the above two definitions, we may easily get an algorithm for how to verify the *α*-connectivity of a generalized uncertain graph as follows.

  Step 1. According to the pre-given confidence level *α*, write out the fundamental subgraph of the generalized uncertain graph *G* about the confidence level *α*.
  Step 2. Write down the adjacency matrix $\bar{A_{G}}$ of the fundamental subgraph of the generalized uncertain graph *G* about the confidence level *α*.
  Step 3. Calculate the value $\bar{R}=I+\bar{A_{G}}+\bar{A_{G}^{2}}\;+\bar{A_{G}^{3}}+\ldots +\bar{A_{G}^{k-1}}$, in which *k* is the order number of the fundamental subgraph of the generalized uncertain graph *G* about the confidence level *α*.
  Step 4. According to Theorem 1, we can easily know that the generalized uncertain graph *G* is *α*-connected if $\bar{R}>0$; otherwise, it is not *α*-connected.

**Example 9 .**

Figure 8 illustrates a 7-order generalized uncertain graph, and the uncertain measure of its every edge is 0.75, 0.64, 0.69, 0.5, 0.3, 0.2, 0.89, 0.85, 0.55, 0.62, 0.26, 0.9, 0.7, and 0.28, respectively, and the uncertain measure of its any vertex is 0.6, 0.9, 0.65, 0.79, 0.95, 0.8, and 0.86, respectively.

Figure 9 presents the fundamental subgraph of *G*, and its confidence level is 0.5 when the confidence level *α* is 0.5. Obviously, it is connected, so the generalized uncertain graph *G* is 0.5-connected.  Figure 10 shows the fundamental subgraph of *G*, and its confidence level is 0.65 when *α* is 0.65. Obviously, the graph in Figure 10 is non-connected. Thus, the generalized uncertain graph *G* is non-connected under the confidence level of 0.65. In the following, we let *α* be 0.8, we can get a connected fundamental subgraph of *G*, and its confidence level is 0.8, as shown in Figure 11. Thus, the generalized uncertain graph *G* is 0.8-connected, but its order is 4.

A major application of *α*-connectivity of generalized uncertain graph is that the user can determine the size of the graph and the reliability measure according to different requirements.

**Definition 14 .**

*α*-connectivity index of generalized uncertain graph *G* is defined as follows:

(40) $$\begin{array}{c} \mu \left(G\right)=\underset{\alpha }{\sup}\left\{\text{the graph }G\text{ is }\alpha -\text{connected}\right\}. \end{array}$$

According to the above discussion, we can easily know the relationship between the *α*-connectivity index and the connectedness index of a generalized uncertain graph.

Assume *G* is a generalized uncertain graph, the *α*-connectivity index of *G* is equal to its connectivity index.

### 4.4. Experimental Verification Analysis

We verify the implementation stability and efficiency of the algorithm about the connectivity index of generalized uncertain graph using a large number of experiments. Without a trusted query algorithm according to the reliability index, conditional connectivity query, and so on, the paper only studies the main query methods in different data set scales and the efficiency of different constraint conditions.

The experimental data are implemented in the operating system of Windows 7, the processor of 1.8GHZ, and the memory of 8G condition, using the artificial simulation in the programming environment of Visual *C*++ 6.0.

In the experiment, we generate randomly some uncertain networks.  Table 1 shows the numbers of vertices and edges in these networks. These edges in every uncertain network are randomly created between the two vertices. The reliability of each uncertain edge is randomly created among the real numbers in [0,1], and the reliability of each uncertain vertex is randomly created among the real numbers in [0,1].

There are two parts in the experiment. In the following part, we will test the credibility of algorithm of connectivity index generalized uncertain graph if there is no limitation. In Experiment 1, we test the change in algorithm performing required time based on the different scales of edges and vertices. We test the time variation of the algorithm execution under the same number of edges in Experiment 2.

**Experiment 1 .**

Figure 12 shows the results of the query results. The execution time of the algorithm has a similar distribution to the change in the number of vertices and edges in the uncertain network.

**Experiment 2 .**

To test the validity of the experiment based on the query algorithm under the user specified the number of edges and vertices in uncertain network.  Figure 13 shows the query results.  Figure 13 shows that it is a similar distribution of the algorithm performing required time, and the change corresponds to a change in the number of edges and vertices in uncertain network.

## 5. Conclusion

A connected graph is the most basic property in classic graph theory. However, in certain actual applications, different uncertain factors are frequently encountered and must be solved. This study puts forward a definition of generalized uncertain graphs and connectivity index and *α*-connectivity of generalized uncertain graphs based on the uncertainty theory and proposes an algorithm for connectivity index and *α*-connectivity by symplectic adjacency matrix of a generalized uncertain graph. This study presents the definition of *α*-connectivity index of generalized uncertain graphs and obtains the relationship between the *α*-connectivity index and the connectivity index of a generalized uncertain graph. In the end, the study employs numerical experiments to verify the correctness of this new algorithm.

## Figures and Tables

**Figure 1:** A 4-order graph.

**Figure 2:** An uncertain 4-order graph.

**Figure 3:** A generalized uncertain 4-order graph.

**Figure 4:** Basic graph of Figure 3.

**Figure 5:** A 2-order generalized uncertain graph.

**Figure 6:** A 3-order generalized uncertain graph.

**Figure 7:** Basic graph of the generalized uncertain graph (G) in Figure 6.

**Figure 8:** Generalized uncertain graph (G) of order 7.

**Figure 9:** An confidence level is 0.5 of fundamental subgraph in Figure 8.

**Figure 10:** An confidence level is 0.65 of fundamental subgraph in Figure 8.

**Figure 11:** The confidence level is 0.8 of fundamental subgraph in Figure 8.

**Figure 12:** Algorithm execution time versus number of edges and vertices.

**Figure 13:** Algorithm execution time versus number of edges and vertices with the reliability constraints (*α*  = 0.5).

**Table 1:** Artificial simulation data of uncertain network.

Name	Vertices	Edges
G1	145	9100
G2	135	7100
G3	125	5100
G4	115	5100
G5	105	4600
G6	95	3600
G7	85	3100
G8	75	2100
G9	65	1800
G10	45	650

## Data Availability

Data sharing is not applicable to this article as no new data were created or analyzed in this study.
